# Electroacupuncture of Weizhong (BL-40) Acupoint Inspires Muscular Satellite Cell Regeneration and Promotes Muscle Repair Capacity after Back Muscle Injury in Sprague-Dawley Rat Model

**DOI:** 10.1155/2022/2695679

**Published:** 2022-08-04

**Authors:** Bi-Xiu Huo, Zhi-Ling Wang, Ying-Qian Jiao, Xiao-Yi Wang, Yan-Li Lang, Yong-Jun Mi, Zhi-Xin Li, Zhi-Zhong Ma

**Affiliations:** ^1^Department of Traditional Chinese Medicine, Chengdu University of Traditional Chinese Medicine, Chengdu 610072, China; ^2^Department of Integration of Traditional Chinese and Western Medicine, School of Basic Medical Sciences, Peking University Health Science Center, Peking University, Beijing 100191, China; ^3^Department of Rehabilitation, Hyogo College of Medicine, Nishinomiya, Hyogo, 6638501, Japan

## Abstract

**Background:**

Back muscle injury is the most common illness involved in aged people. Muscular satellite cells, playing a key role in the muscle repairing process, are gradually losing their regenerative ability with aging, which attenuates the injured muscle repairing process. Electroacupuncture at Weizhong acupoint has been widely used in the treatment of young and aged patients with back muscle damage. Its efficacy has been proven by a randomized double-blind placebo clinical trial. However, the rehabilitation mechanisms are largely unknown. This study will explore the possible mechanisms associated with electroacupuncture at the Weizhong acupoint (BL 40) promoting muscle repairing ability.

**Method:**

A total of 58 male and female Sprague-Dawley rats were divided into a younger group (4-month-old) and an aged group (16-month-old), younger and aged rats were further divided as a sham, injured, injured rats treated with electroacupuncture at Weizhong point or treated with Non-Weizhong point groups. The back muscle injury model was produced in rats as a previously described method with modification. Furthermore, Weizhong acupoints underwent electroacupuncture treatment with 15 V magnitude, 2 Hz/10 Hz frequency density, 1.0 mA current intensity, and 10 min each day for 10 consecutive days using HANS's electroacupuncture apparatus. After the last treatment, the paravertebral muscles and serum of all animals were undergone histological, immunohistochemistry, and flow cytometry analysis. Serum levels of Creatine Kinase (CK) and proinflammatory cytokine, interleukin 6 (IL-6), were measured separately by using ELISA kit.

**Results:**

Electroacupuncture of Weizhong (BL 40) acupoints significantly attenuated back muscle damage in both young and aged rats, increasing PAX7 (a marker of muscle satellite cells) and MYOD (major marker of myoblasts) cells, simultaneously, reducing serum proinflammatory cytokines, IL-6, and downregulation of p38 MAPK signaling in aged muscular satellite cells.

**Conclusion:**

Our studies suggest that electroacupuncture of Weizhong (BL 40) acupoints can restore aged back muscular satellite cells and their regeneration capacity. These suggested electroacupuncture may be a potential means of promoting rehabilitation for muscular injury in aged patients.

## 1. Introduction

Muscle injury, including back muscle injury, is the most common injury in daily clinical cases [1–3]. Clinically, muscle damages are more aggravated with aging, which become increasingly one of the main conditions causing disability in the elderly [4, 5]. At present, the primary treatment for this disease is the application of nonsteroidal anti-inflammatory drugs (NSAID), which temporarily relieve the pain [6]. However, muscle injury often happens and is more likely to cause an accumulation of damage, thus it is frequently referred to clinically as repetitive strain injury (RSI) [7] or cumulative trauma disorders (CTDs) [8]. Long-term use of NSAIDS may cause severe side effects in patients, especially elderly patients, such as gastrointestinal bleeding [9]. Therefore, to investigate better therapeutic methods, which not only relieve pain but also simultaneously strengthen rehabilitation, present clinical benefits for elderly patients' health conditions, and improve their quality of life [10].

In fact, the skeletal muscle itself retains a high capacity to repair its damages. Previous studies have demonstrated that satellite cells (SC), i.e., muscular stem cells, play a central role in the process of muscle regeneration and repair [11]. In normal physiological conditions, this subset of cells remains in a quiescent state. Once the muscle is exposed to injury, muscular satellite cells are activated rapidly to expand and proliferate [12]. Most activated cells then differentiate into myoblasts accompanied by high expression of myoblast determination protein (MYOD). These myoblasts are further differentiated into mononuclear myocytes, which can fuse with each other or with damaged myofibers, to repair the injured muscles [13]. Recent studies have confirmed that transcription factors paired box 7 (PAX7) are critical to maintaining the quiescence of SC in normal conditions while undergoing self-renewal, proliferation, and differentiation in injured conditions; therefore, PAX7 positive cells are indispensable for the efficient repair of muscle after injury [14, 15].

During aging, muscular repair declines and the skeletal muscle undergoes atrophy or sarcopenia progressively [16]. Studies have displayed that age-related proliferation and self-renewal dysfunction of SCs is the principal pathogenic reasons causing impaired muscle repair in age-related muscle wasting diseases [4, 17]. Both microenvironment factors and cell-intrinsic factors have been demonstrated to impact the regenerative capacity of SCs severely [18]. These studies suggest that enhancing the regenerative capacity of muscle stem cells may promote muscle repair in elderly patients following the injury.

Acupuncture including acupuncture at Weizhong acupoint, one type of traditional Chinese therapy, has been used in treatments of chronic low back pain [19], muscle damage or atrophy caused by traumatic injury, cerebral stroke [20, 21], or spinal cord injury [22], and showed obvious recovery effects in function. The effectiveness of electroacupuncture on muscle pain, demonstrated by multiple randomized controlled clinical trials in many countries and China, has been reported [19, 23]. Recent clinical studies show that electroacupuncture can effectively alleviate elderly patients with low back muscle pain, with the rate for relieving chronic pain is 40.6% [24]. Animal studies show that electroacupuncture could enhance the muscle repair processes after injury in aged rats or mice, but the underlying mechanisms have not yet been clarified. In this study, our main purpose is to explore the mechanism whether electroacupuncture could affect aged muscular satellite cell regenerative capacity by intervening intracellular or environmental factors around MuSC. Since Weizhong (BL-40) acupoint is the most commonly used acupoint in the treatment of post-stroke sarcopenia or chronic back pain in clinical practice, in these studies, we produce the back muscle injury rat model to test if electroacupuncture can promote the repair process in young and aged rats. We believe the elucidation of these problems will help us better understand the mechanism of acupuncture to boost the injury repair ability of the elderly.

## 2. Materials and Methods

### 2.1. Animals

Male and female Sprague-Dawley (SD) rats, including younger rats (4-month-old) and aged rats (16-month-old), were obtained from the Animal Center of Peking University (certificate no. SCXK (Jing) 2006-0011). The rats were raised in cages at a temperature of 22 ± 2°C and relative humidity of 40 ± 5% under a 12-hour light/dark cycle, with a standard diet and water ad libitum. The investigations complied with the Guide of the Peking University Animal Research Committee. The experimental protocols were approved by Peking University Biomedical Ethics Committee Experimental Animal Ethics Branch (Approved number: LA2018-045).

### 2.2. Major Instruments and Regents

Hans' Electroacupunture apparatus (Catalog No. hans-200a/100b, Beijing, China)，is a kind of small portable electroacupuncture instrument approved for using for treating patients, or used as a tool in research studies. The primary antibodies, including the anti-MYOD antibody (ab203383), anti-PAX7 antibody (ab187339), and anti-p38 MAPK (mitogen-activated protein kinases) (sc-166182), were purchased from Santa Cruz Biotechnology, Inc., Company (Oregon, USA) and diluted at 1 : 1000 when used. The secondary antibody, Goat Anti-Rabbit IgG H&L (FITC) (ab6717), was purchased from Abcam Company (Cambridge, MA 02139-1517, USA).

### 2.3. Experimental Grouping and Back Muscle Injury Model Making

SD rats were first separated into the following groups based on age, gender, and treatment. (1) YS: young sham group (4-month-old, *n* = 8; four males and four females); (2) YI: young injured group (4-month-old, *n* = 7; four males and three females); (3) YI + WZ: young injured rats treated with electroacupuncture of Weizhong (BL-40) acupoint (4-month-old, *n* = 7; four males and three females); (4) YI + NWZ: young injured rats treated with electroacupuncture of Non-Weizhong (BL-40) acupoint (4-month-old, *n* = 7; four males and three females); (5) AS: aged sham group (16-month-old, *n* = 8; four males and four females); (6) AI: aged injured rats (16-month-old, *n* = 7; four males and three females); (7) AI + WZ: aged injured rats treated with electroacupuncture of Weizhong (BL-40) acupoint (16-month-old, *n* = 7; four males and three females); (8) AI + NWZ: aged injured rats treated with electroacupuncture of Non-Weizhong (BL-40) acupoint (16-month-old, *n* = 7; four males and three females).

“The back muscle injury model was produced in SD rats as a previously described method with modification [25–27]. Briefly, each animal was administered ibuprofen (SK&F) orally for postoperative pain relief (15 mg/kg), and once again at 12 hours after surgery (twice a day). About 30 minutes later, each animal has been anesthetized with isoflurane inhalation. Then, the right and left sides of the paravertebral muscle are subjected to crushing to approximately 500 g/cm^2^ force for 2 minutes, once a day for 5 days. It has been proved in our preliminary experiment that the repeated crush with such intensity and duration could cause the obvious back muscle repetitive injuries. In the sham group, only the back skin of rats is stretched. In our preliminary study, this group underwent the same anesthesia process as the model group and the treatment group but without muscle damages.”

### 2.4. Electro-Electroacupuncture

Rats were placed in a prone position in a custom-built rat stationary holder and immobilization was ensured. Both hind legs were secured out of the holder box. After lying, prostrate quietly for 10 min without any external stimulus. The area of electroacupuncture points was disinfected with medical alcohol. Each of The bipolar needle electrodes was inserted about 5.0 mm from the Weizhong point or non-Weizhong point, which is about 5.0 mm away from the accurate point of Weizhong (Electroacupuncture needle specification 0.16 mm × 10 mm). For all protocols, electroacupuncture points were stimulated at 15 V magnitude, the density wave was 2 Hz/10 Hz frequency, 1.0 mA current intensity, and 10 min each day by using Hans's electroacupuncture apparatus (HANS-200A/100B. Beijing, China), treatment for 10 Days. The lower limbs appeared slightly trembling to prevail. At the end of the treatment, the acupoints were sterilized in alcohol and put back in the rat box.

### 2.5. Animal Anesthesia and Blood Collection

After the last electroacupuncture, the animals were anesthetized with pentobarbital (30 mg/kg, intraperitoneal injection), and the blood was collected from the aorta after anesthesia in rats using a non-heparinized blood collection tube. Until clots, the blood was centrifuged with a desktop centrifuge (Eppendorf, Germany) at 3000 rpm for 15 min. The supernatant serum was stored at −20°C to measure the serum level of Creatine kinase (CK) and proinflammatory cytokine, Interleukin 6 (IL-6).

### 2.6. Animal Sacrifice and Tissue Harvesting

After the collection of blood, the experimental animals were immediately euthanized by decapitation. The euthanasia procedures were consistent with the American Veterinary Medical Association (AVMA) Guidelines. Then one side of the paravertebral back muscles and spinal cord were dissected and fixed with 4% paraformaldehyde in 0.1 M phosphate buffer (PBS) and dehydrated with 30% sucrose solution in 0.1 M PBS.

### 2.7. Histological Staining

For histological staining, parts of each animal's back muscles were embedded with paraffin and cut at 10 *μ*m thickness, and stained with Hematoxylin-Eosin (H-E staining).

### 2.8. Immunohistochemistry Staining

After fixation and dehydration in 30% sucrose phosphate buffer, parts of each animal's back muscles were embedded with embedding medium (OCT, SAKURA, USA) and cut at 20 *μ*m thickness frozen section with a microtome. Then, the sections were incubated successively with primary antibodies, Anti-MYOD antibody (Abcam, 1 : 1000), Anti-p38 MAPK (sc-1661821 : 1000), the secondary antibody, goat biotinylated conjugated polyclonal anti-rabbit antibody (1 : 250; Vector Laboratories), and horseradish-peroxidase-conjugated avidin-biotin complex (Vector Laboratories). Sections were then exposed to diaminobenzidine (DAB) for detection. To adequately quantify MYOD and p38 MAPK positive cells, we used the nuclear counterstain methyl green (Vector Laboratories) and counted MYOD and p38 MAPK positive cells.

### 2.9. Isolation of Muscle Stromal Cells and Flow Cytometry Analysis

Muscle stromal cells (containing satellite cells) were isolated, as described previously, with modifications [28, 29]. Briefly, portions of the back muscles of rats were minced under a dissection microscope and enzymatically digested with 0.2% Collagenase Type I solution (Worthington Biochemical, Lakewood, NJ) in DMEM at 37°C for 30 min, and 0.25% Trypsin-EDTA for 15 min, the cell suspension was filtered through a 40 *μ*m nylon filter (BD Biosciences). The suspended cells were cultured in 6-well plates with DMEM supplemented with 10% FBS (Invitrogen), and 1.0% penicillin-streptomycin for 24 hours. The isolated cells were then fixed and perforated with fixation and permeabilization solution (BD Biosciences). Then, the isolated cells were incubated with FITC labeled Anti-PAX7 antibody (Abcam) and underwent flow cytometry analysis (FACS Calibur™, BD Biosciences). The PAX7 positive cells were quantified.

### 2.10. Serum Level of Creatine Kinase (CK) and Proinflammatory Cytokine, Interleukin 6 (IL-6)

The levels of IL-6 in serum were determined by using IL-6 ELISA Kit (Ex-Cell Biology, Shanghai, China) according to the manufacturer's instructions. The levels of Creatine kinase (CK) were determined by using the Beckman Coulter AU2700 Chemistry Analyzer.

### 2.11. Statistical Analysis

All parameters were expressed as mean ± S.D. By using the software GraphPad Prism 9, statistical analysis was performed using one-way ANOVA followed by Student's *t* test assuming two-tailed distributions. *P*-value less than 0.05 was statistically significant. By using the software SPSS 20, the Chi-square test was performed for pathological imaging analysis and was used for multivariate statistical analysis.

## 3. Results

### 3.1. Electroacupuncture of Weizhong (BL-40) Acupoints Can Significantly Decrease Back Muscle Injury in Both Young and Aged Rats

As shown in Figure 1, histological examination indicates that the back muscle in both young and aged rats appeared with visible damage after being injured. Some myofibers have been lacerated. The interstitial area was infiltrated by inflammatory cells and edema appeared as indicated by the expanded extracellular space. In both young and aged rats, after damage, the stromal cells, including fibroblasts and satellite cells, were more crowded near the nuclei of the myofibers. (*P* < 0.05, young sham (YS) vs. young injured (YI), aged sham (AS) vs. aged injured (AI) group, with Chi-square test). Serum creatine kinase (CK), which is released from the damaged muscle, also increased dramatically in both YI and AI groups (YI vs. YS and AI vs. AS group, one-way ANOVA followed by Student's *t*-test).

After electroacupuncture of the Weizhong acupoint, myofibers' cellular integrity the arrangement in both young and aged rats were restored clearly. Interstitial edema shrunk as the extracellular space is becoming narrowing. Interstitial cell density is becoming increasing. (*P* < 0.05, YI + WZ vs. YI, and AI + WZ vs. AI group, with Chi-square test).

While electroacupuncture at the non-Weizhong point, the rats showed no notable effects when compared with the Weizhong acupoint treatment group. See Figure 1 for details.

### 3.2. Electroacupuncture of Weizhong (BL-40) Acupoints Significantly Increased the Number of Myoblast Determination Protein (MYOD) Positive Satellite Cells in the Back Muscle of Young and Aged Injured Rats

To achieve the repair of muscle injury, the satellite cells must differentiate into myoblasts, which further transform into mononuclear myofibers, fusing with damaged myofibers to repair the damaged muscle. During differentiation of myoblasts, myoblast determination protein (MYOD) was upregulated in the cells. Therefore, MYOD is used as the key biomarker linked with the muscle repair process [13, 18].

As shown in Figure 2, after injured MYOD, positive cells in both young and aged groups are clearly increased. After electroacupuncture of Weizhong (BL-40) acupoints, MYOD positive cells in either young or aged rats are further increased dramatically significantly (^ϯϯϯ^*P* < 0.001, YI vs. YS, AI vs. AS, ^##^*P* < 0.01, YI + WZ vs, YI, AI vs. AI + WZ, one-way ANOVA followed by using Student's *t*-test). While stimulating the non-Weizhong acupoint, no statistically significant changes in myoblast numbers were displayed.

When the aged group was compared with the young group, MYOD positive cells decreased significantly, which indicated the muscular repair capacity in the aged group declined, while electroacupuncture of Weizhong acupoint can restore the capacity (*P* < 0.001, VS. YS, *P* < 0.01, AI + WZ vs. AI, one-way ANOVA followed by using Student's *t*-test). These results indicate electroacupuncture of Weizhong promotes differentiation from satellite cells to MYOD positive myoblasts, which play a critical and indispensable role in muscle repair.

### 3.3. Electroacupuncture of Weizhong (BL-40) Acupoints Significantly Increased the Number of PAX7 Positive Satellite Cells in the Back Muscle of Aged and Young Injured Rats

Previous studies have shown that MYOD expression is regulated by PAX7 after birth. Recent studies have shown that PAX7 plays a key role in maintaining muscle satellite cell homeostasis in adult or aged people [30]. The purpose of this study is to figure out whether the changes of PAX7 positive cells appeared in young and old rats after muscle injury, and whether electroacupuncture treatment will intervene with these changes.

As shown in Figure 3, our results showed that the number of PAX7 positive cells in the aged rats decreased significantly compared with the young rats (*P* < 0.05, VS. YS). After injury, the number of PAX7 positive cells showed mildincreasing (*P* < 0.01, YI vs. YS, *P* < 0.05, AI vs. AS). After treatment with Weizhong electroacupuncture, the number of PAX7 positive cells in both young and aged groups increased significantly (*P* < 0.01, YI + WZ vs. YI, *P* < 0.001, AI + WZ vs. AI). Electroacupuncture on non-Weizhong acupoint may also increase the PAX7 positive cells significantly (*P* < 0.001, AI + NWZ vs. AI), but much weaker than treatment on Weizhong acupoint (*P* < 0.01, AI + NWZ vs. AI + WZ).

These results indicate the pool of PAX7 positive cells in aged rats is shrunken, whereas electroacupuncture on Weizhong acupoint represents recovery effects to preserve the number of satellite cells in aged rats.

### 3.4. Electroacupuncture Weizhong (BL-40) Acupoints Significantly Decreased the p38*α*/*β* MAPK (Mitogen-Activated Protein Kinase) Positive Cell Numbers of Back Muscle of Young and Aged Injured Rats

Recent studies demonstrate that p38*α*/*β* MAPK (mitogen-activated protein kinase) expression in SC increases with aging, which may cause permanent cell cycle exit and cell arrest, which limit the expansion of satellite cells, inhibiting the regeneration capacity of aged muscle stem cells.

As shown in Figure 4, our results showed that p38*α*/*β* MAPK positive cell numbers increased in old injured rats compared with yang injured rats dramatically (*P* < 0.01, AI vs. YI). After electroacupuncture treatment, p38*α*/*β* MAPK expressions were suppressed remarkably in both young and aged injured rats (*P* < 0.05, YI + WZ vs. YI, *P* < 0.05, AI + WZ vs. AI). These suggested p38*α*/*β* MAPK to injury is heightened in both yang and aged rats, while electroacupuncture can downregulation of p38 MAPK signaling, which may restore the proliferation and differentiation capacity of aged muscle stem cells in back muscle post-injury.

### 3.5. Electroacupuncture of Weizhong (BL-40) Acupoints Significantly Reduced Proinflammatory Cytokine, IL-6 in the Serum of Young and Aged Injured Rats

IL-6 is a proinflammatory cytokine increased when body tissue is damaged and aging. As an upstream factor of p38 MAPK signaling, secretion of proinflammatory cytokines by macrophages suppresses PAX7 expression and induces satellite cell cycle arrest [12].

As shown in Figure 5, after being injured, serum level of IL-6 was heightened prominently in both young and aged rats (*P* < 0.001, YI vs. YS, AI vs. AS, one-way ANOVA followed by using Student's *t*-test). In aged sham rats, IL-6 levels also increased more evidently than in young sham rats (*P* < 0.05). Electroacupuncture of Weizhong acupoint was able to lower the serum IL-6 level dramatically (*P* < 0.001, YI + WZ vs. YI, AI + WZ vs. AI, one-way ANOVA followed by using Student's *t*-test). These results indicate electroacupuncture possesses effects to lower the inflammatory conditions around the satellite cells.

## 4. Discussion

Our results demonstrate that electroacupuncture of Weizhong (BL-40) acupoint presents significant recovery effects on back muscle damage in both young and aged rats. Simultaneously, electroacupuncture of Weizhong is also able to promote the muscle repair process evidenced by increasing MYOD positive myoblasts formation, which plays a critical role to fuse with damaged myofibers hereby to repairing the damaged muscles. As the progenitors of MYOD myoblasts, PAX7 positive cells were declined in aged rats and restored by electroacupuncture of Weizhong acupoint. To investigate the mechanisms for rehabilitation effects of electroacupuncture at the Weizhong acupoint, we identified the electroacupuncture downregulation of p38 MAPK signaling in muscular satellite cells. Additionally, IL-6 pro-inflammatory cytokine in SC's niche secreted by macrophages, which are accumulated when the muscle is injured, is reduced by electroacupuncture of the Weizhong acupoint. Our results revealed that electroacupuncture could enhance muscle repair after injury in both young and aged rats, and restore aged muscular satellite cell regeneration capacity by intervening with proinflammatory cytokines, IL-6, p38 MAPK signaling, PAX7, and MYOD expression. Our results provide evidence that electroacupuncture could be method applied to boost muscle repair in aging and injury.

Muscle repairs rely on satellite cell numbers and functions including self-renew and differentiation. When a muscle is damaged, SCs are rapidly differentiated into myoblasts and myocytes, which fuse with damaged myofibers hereby to repair muscle damage. MYOD is a featured biomarker of myoblasts and mononuclear myocytes. MYOD gene expression is increased remarkably after muscle injury [13, 30]. Thus, amplification of MYOD-positive cells indicates the differentiated capacity of SC is strengthened. In our study, electroacupuncture of Weizhong acupoint can increase the number of MYOD positive cells. This suggested the SC differentiating ability is stimulated and muscle repair accelerated. This result is consistent with the results of clinical studies, which show electroacupuncture can accelerate the recovery process among patients with a muscle injury, and post-stage stroke or paralysis [31, 32].

MYOD positive cells are derived from PAX7 positive satellite cells. PAX7 positive cells have also undergone expansion by self-renewal mode, by which the SC pool is replenished in Pax7 positive satellite cells in order to cope with next muscle damages afterward [13, 33]. Until now, a lot of research has been done on satellite cells. Using fluorescence-activated cell sorting (FACS) technology, the Pax7-expressing population has been isolated and characterized by various combinations of antibodies including CD34, *α*7-integrin, *β*1-integrin, syndecan-4, VCAM-1, and CXCR4. [28]. The role of these cell surface biomarkers in satellite cell fate required further studies, whereas Pax7 is approved as a critical and indispensable transcriptional regulatory factor in determining the quiescence and self-renewal ability of satellite cells.

In our study, we used anti-PAX7 antibody directly quantified PAX7 positive satellite cells. Our results indicate PAX7 positive cells are decreased notably after muscle injury in young rats, which suggests the satellite cells have undergone differentiation, thus the satellite cell pool is temporarily contracted. In aged rats, PAX7 positive cells sharply cut down in the back muscle of aged rats, while electroacupuncture of Weizhong acupoint increased these populations of cells significantly. These suggested that electroacupuncture could restore self-renewal function. These results are concordant with the results of the clinical observations that age-related atrophic conditions could be improved by electroacupuncture.

PAX7 satellite cells declined mainly from both intrinsic and micro-environmental factors [18]. During aging, the molecules in the satellite cells undergo repeated injury from free radical, oxygen species, inflammation factors, etc. Recent studies demonstrated that p38a/B MAPK signaling in SC increased with aging, which may cause permanent cell cycle exit and cell arrest, which limit the expansion of satellite cells, and weaken the regeneration capacity of aged muscle stem cells, while neutralization of p38 MAPK with p38 MAPK chemical inhibitors strongly improve stem cell engraftment in severe muscular pathologies and restore regenerative capacity in aging individuals.

Among many factors, proinflammatory cytokines, IL-6, one of the key upstream factors that activate p38MAPK, heightened dramatically in the aged and injured. After the injury, the accumulated macrophages secreted a great quantity of IL-6. By activating JAK/STAT3, IL-6 may cause muscle satellite cells to undergo terminal differentiation, instead of expansion. Thus, the satellite cell pool is minimized or exhausted with aging and repeated injury.

Following electroacupuncture, the elevated level of IL-6 in aged animals decreased, thereby avoiding the loss of satellite cells, which retain the homeostasis of satellite cells with aging, which is critical in the repair of future injuries. Our results indicate electroacupuncture possesses effects to lower the inflammatory conditions around the satellite cells. These results are consistent with the results of the clinical observations that electroacupuncture presents obvious effects on inflammatory conditions in muscle and other soft tissues [34, 35].

## 5. Conclusion

In conclusion, our study demonstrated that electro-electroacupuncture at Weizhong (BL-40) acupoints can significantly reduce back muscle damage in young and aged rats, enhancing satellite cell differentiation and self-renewal capacity, therefore, strengthening muscle repair. To improve both intrinsic and extrinsic niche factors that cause satellite cell senescence, electroacupuncture can preserve and restores the muscle regenerative ability in young and aged rats. Certainly, further studies are required. This study provides evidences supporting electroacupuncture as a practical way to inspire innate muscle repair in young and aged patients.

## Figures and Tables

**Figure 1:** Electroacupuncture of Weizhong (BL-40) acupoints significantly decreased the damage to back muscle in young and aged rats. (a) Representative images of H&E staining of the back muscles of rats of the following groups. YS: young sham group (*n* = 8); YI: young injured group (*n* = 7); YI + WZ: young injured group treated with electroacupuncture of Weizhong (BL-40) acupoint (*n* = 7); YI + NWZ: young injured group treated with electroacupuncture of Non-Weizhong (BL-40) acupoint (*n* = 7); AS: aged sham group (*n* = 8); AI: aged injured group (*n* = 7); AI + WZ: aged injured group treated with electroacupuncture of Weizhong (BL-40) acupoint (*n* = 7); AI + NWZ: aged injured group treated with electroacupuncture of Non-Weizhong (BL-40) acupoint (*n* = 7); The electroacupuncture last for 10 days after the rat back muscle injured for 5 days. Scale bar: 50 *μ*m. (b) Quantification analysis of average serum CK level of all rats (*n* = 8 in young sham and aged sham groups, *n* = 7 in other groups). All data are represented as the mean ± SD. Student's *t*-test was used for all statistical analyses (^ϯϯϯ^*P* < 0.001,^#^*P* < 0.05,^##^*P* < 0.01).

**Figure 2:** Electroacupuncture of Weizhong (BL-40) acupoints significantly promotes myoblast determination protein (MYOD) of back muscle in young and aged rats. (a) Representative images of MYOD immunohistochemically staining of the back muscles of rats in the following groups, YS: young sham group (*n* = 8); YI: young injured group (*n* = 7); YI + WZ: young injured rats treated with electroacupuncture of Weizhong (BL-40) acupoint (*n* = 7); YI + NWZ: young injured rats treated with electroacupuncture of non-Weizhong (BL-40) acupoint (*n* = 7); AS: aged sham group (*n* = 8); AI: aged injured rats (*n* = 7); AI + WZ: aged injured rats treated with electroacupuncture of Weizhong (BL-40) acupoint (*n* = 7); AI + NWZ: aged injured rats treated with electroacupuncture of non-Weizhong (BL-40) acupoint (*n* = 7); The electroacupuncture last for 10 days after the rat back muscle injured for 5 days. Scale bar, 100 *μ*m. The red arrow in the figures points to MYOD-positive cells. (b) Quantification analysis of average MYOD positive cell number of all rats (*n* = 8 in young sham and aged sham groups, *n* = 7 in other groups). All data are represented as the Mean ± SD. Student's *t*-test was used for all statistical analyses (^ϯϯϯ^*P* < 0.001,^#^*P* < 0.05,^##^*P* < 0.01).

**Figure 3:** Electroacupuncture of Weizhong (BL-40) acupoint significantly increased PAX7 positive cells. (a) Representative images of FITC labeled PAX7 flow cytometry analysis of the back muscle of the following groups. YS: young sham group (*n* = 8); YI: young injured group (*n* = 7); YI + WZ: young injured rats treated with electroacupuncture of Weizhong (BL-40) acupoint (*n* = 7); YI + NWZ: young injured rats treated with electroacupuncture of Non-Weizhong (BL-40) acupoint (*n* = 7); AS: aged sham group (*n* = 8); AI: aged injured rats (*n* = 7); AI + WZ: aged injured rats treated with electroacupuncture of Weizhong (BL-40) acupoint (*n* = 7); AI + NWZ: aged injured rats treated with electroacupuncture of Non-Weizhong (BL-40) acupoint (*n* = 7). The electroacupuncture may last for 10 days after the rat back muscle is injured for 5 days. Scale bar, 100 *μ*m. (b) Quantification analysis of average PAX7 positive cells of all rats (*n* = 8 in young sham and aged sham groups, *n* = 7 in other groups). All data are represented as the Mean ± SD. The student's *t*-test was used for all statistical analyses (^ϯϯϯ^*P* < 0.001,^###^*P* < 0.001,^##^*P* < 0.01).

**Figure 4:** Electroacupuncture Weizhong (BL-40) acupoints significantly decreased the p38*α*/*β* MAPK (mitogen-activated protein kinase) positive cell numbers of the back muscle of young and aged injured rats. (a) Representative images of p38*α*/*β* MAPK immunohistochemistry staining of the back muscles in the following groups. YS: young sham group (*n* = 8); YI: young injured group (*n* = 7); YI + WZ: young injured rats treated with electroacupuncture of Weizhong (BL-40) acupoint (*n* = 7); YI + NWZ: young injured rats treated with electroacupuncture of non-Weizhong (BL-40) acupoint (*n* = 7); AS: aged sham group (*n* = 8); AI: aged injured rats (*n* = 7); AI + WZ: aged injured rats treated with electroacupuncture of Weizhong (BL-40) acupoint (*n* = 7); AI + NWZ: aged injured rats treated with electroacupuncture of non-Weizhong (BL-40) acupoint (*n* = 7). The electroacupuncture may last for 10 days after the rat back muscle is injured for 5 days. Scale bar, 50 *μ*m. (b) Quantification analysis of average p38*α*/*β* MAPK positive cells in rats (*n* = 8 in young sham and aged sham groups, *n* = 7 in other groups). All data are represented as the Mean ± SD. Student's *t*-test was used for all statistical analyses (^ϯ^*P* < 0.05,^##^*P* < 0.01,^###^*P* < 0.001).

**Figure 5:** Electroacupuncture of Weizhong (BL-40) acupoints significantly decreased serum proinflammatory cytokine, IL-6 levels in aged rats. (a) Quantification analysis of average serum interleukin 6 levels of all rats in the following groups. YS: young sham group (*n* = 8); YI: young injured group (*n* = 7); YI + WZ: young injured rats treated with electroacupuncture of Weizhong (BL-40) acupoint (*n* = 7); YI + NWZ: young injured rats treated with electroacupuncture of non-Weizhong (BL-40) acupoint (*n* = 7); AS: aged sham group (*n* = 8); AI: aged injured rats (*n* = 7); AI + WZ: aged injured rats treated with electroacupuncture of Weizhong (BL-40) acupoint (*n* = 7); AI + NWZ: aged injured rats treated with electroacupuncture of non-Weizhong (BL-40) acupoint (*n* = 7). The electroacupuncture may last for 10 days after the rat back muscle is injured for 5 days. All data are represented as the Mean ± SD. Student's *t*-test was used for all statistical analyses (^ϯϯϯ^*P* < 0.001,^##^*P* < 0.01).

## Data Availability

The datasets generated during and/or analyzed during the current study are available from the corresponding author on request.
